# Efficacy and Safety of Vitamin D Adjuvant Therapy for Ulcerative Colitis: A Meta-Analysis

**DOI:** 10.1155/2022/6836942

**Published:** 2022-07-20

**Authors:** Xinyi Guo, Changxing Liu, Yahui Huang

**Affiliations:** ^1^First School Clinical Medicine, Shaanxi University of Traditional Chinese Medicine, Xianyang 712046, China; ^2^Xi'an Traditional Chinese Medicine Hospital, Xi'an 710016, China

## Abstract

**Objective:**

To examine the clinical efficacy and safety of Vitamin D in the treatment of ulcerative colitis in a systematic manner.

**Methods:**

RCT studies on Vitamin D in the treatment of ulcerative colitis were searched from CNKI, Wanfang Data, PubMed, Cochrane Library, and Web of Science databases. RevMan 5.4 software was used for analysis.

**Results:**

10 articles were included, including 1077 patients. Meta-analysis results showed that when clinical efficacy was used as the outcome index, the clinical efficacy of the oral vitamin group was higher than that of the conventional treatment group (OR = 4.07, 95% CI 2.64-6.27), and the difference was statistically significant (*Z* = 6.38, *P* < 0.00001). When the Mayo risk score was used as the outcome index, the difference was statistically significant, indicating that oral Vitamin D significantly reduced the Mayo risk score (MD: -0.41, CI = (−0.47, −0.34), *Z* = 13.09, *P* < 0.00001). Using the intestinal mucosal barrier as the outcome index, the results showed that (1) the MDA group (MD = −0.75, 95% CI (-0.96~-0.53), *P* < 0.00001), (2) the DAO group (MD = −1.17, 95% CI (-1.39-0.95), *P* < 0.00001), and the Vitamin D group could effectively improve intestinal mucosal barrier function after sensitivity analysis (MD = −1.00, 95% CI (-1.08-0.92), *P* < 0.00001). When inflammatory factors were used as outcome indicators, IL-6, TNF-*α*, and CRP groups had statistical significance (MD = −4.50, 95% CI (-5.13-3.87), *P* < 0.00001); MD = −7.27, 95% CI (18.96-5.58), *P* < 0.00001; and MD = −1.49, 95% CI (-1.76~-1.23), *P* < 0.00001, respectively). When the incidence of adverse reactions was used as the outcome indicator (OR = 0.73, 95% CI (0.34-1.32), *P* = 0.23), there was no significant difference between the two groups.

**Conclusion:**

Vitamin D combined with mesalazine is effective in the treatment of ulcerative colitis, by improving the Mayo score and intestinal barrier function, and reducing inflammatory factors, with no significant safety difference. However, due to the quality of the included researches, more RCT researches needed to provide sufficient evidence to support clinical application. This study is registered with INPLASY 202250044.

## 1. Introduction

Ulcerative colitis (UC) is an inflammatory colonic disease with unknown etiology, characterized by continuous and diffuse colonic mucosal inflammation, commonly manifested as abdominal pain, mucus, pus, blood and stool, etc. [1]. This disease has the characteristics of long course, easy recurrence, and difficult to cure. About 20% of patients with chronic UC have the risk of developing colorectal cancer, and the number of UC cases in China is increasing at present [2]. Western medicine treatment mainly adopts protection and repair of intestinal mucosa, reduction of inflammatory factors, and prevention and treatment of complications. Aminosalicylic acid preparation is the most commonly used drug. If aminosalicylic acid treatment effect is not good, glucocorticoids and immunosuppressants can be added [3].

Mesalazine is the most generally prescribed amino salicylic acid preparation for the treatment of UC, and it helps to protect the mucosa of the intestine. However, mesalazine alone has a low efficacy and a significant rate of side effects in some people [4]. As one of the sterols, Vitamin D is a recognized new immune factor, which exists in the form of 1, 25-hydroxyvitaminD3 (1,25-(OH) D3) in the human body and participates in various autoimmune regulations [5]. Relevant studies have shown that Vitamin D level is negatively correlated with the risk of UC [6], but rigorous and standardized clinical evidence is still lacking. As a result, by examining domestic and international clinical randomized controlled studies on the treatment of UC, this research analyzed the efficacy of Vitamin D on UC and presented evidence-based evidence for the selection of UC treatment plans.

The paper is organized as follows: the data and methods are presented in Section 2.  Section 3 discusses the experiments and results.  Section 4 consists of the discussion, and finally, in Section 5, the research work is concluded.

## 2. Data and Methods

### 2.1. Retrieval Strategy

Figure 1 depicts the article screening procedure. PubMed, Cochrane Library, and Web of Science databases were searched for the “randomised controlled study” using terms like “inflammatory disease”, “Vitamin D”, “mesalazine”, and “Ulcerative colitis”, linked with “AND”/“OR” operators. Chinese search terms such as “ulcerative colitis”, “vitamin D”, “mesalazine”, and “clinical controlled trial” were searched in CKNI, and Wanfang databases.

### 2.2. Inclusion and Exclusion Criteria

#### 2.2.1. Literature Inclusion Criteria

The literature should be a clinical randomized controlled study (RCT study).

#### 2.2.2. Intervention Measures

Vitamin D and mesalazine were given orally to the treatment group, while mesalazine was given alone to the control group.

#### 2.2.3. Efficacy Evaluation Indicators

Refering to Consensus on Diagnosis and Treatment of Ulcerative Colitis by Integrated Chinese and Western Medicine(2017) [7], clinical curative effect is the main indicator..

Secondary indicators are Mayo score, intestinal mucosal function (serum MDA and DAO), inflammatory factors (IL-6, CRP, and TNF-*α*), and incidence of adverse reactions.

#### 2.2.4. Exclusion Criteria

Animal studies, pharmacological studies, or literature with repeated discussions, reviews, and conference summaries and incomplete outcome indicators was excluded.

### 2.3. Data Collection and Extraction

According to the inclusion and exclusion criteria, the two researchers independently screen the title, abstract, and full text of the paper. If there is a dispute on the inclusion or exclusion of the research, all the research members participate in the discussion and make a decision together. Data were extracted from a uniform data extraction table, including first author, publication year, number of cases, sex, evaluation age, intervention, outcome measures, and randomization. A total of 10 RCT studies were included [8–17], with a total of 1077 patients. The basic characteristics are shown in Table 1.

### 2.4. Quality Analysis of Included Literature

The methodological quality of all included RCTs was evaluated using the risk bias assessment tool in the Cochrane Review Manual [18], including (1) whether to use random numbers or computer randomization, (2) whether to implement the allocation hiding scheme, (3) whether blind method is used correctly, (4) data integrity, (5) selective outcome report, and (6) other sources of bias. The risk of bias from included studies is shown in Figure 2.

### 2.5. Statistical Methods

Meta-analysis was conducted using RevMan 5.4 software, and the main effect values were as follows: weighted standard deviation (WMD), standard mean difference (SMD), and 95% credibility interval (CI). If *P* > 0.05 and *I*^2^ ≤ 50%, the fixed effects model could be selected, indicating statistical homogeneity of subjects. On the contrary, if *P* < 0.05 and *I*^2^ > 50%, it indicates that there is heterogeneity in the selected research object, and sensitivity analysis should be conducted step by step by eliminating all studies [19].

## 3. Results

### 3.1. Outcome Index Analysis

#### 3.1.1. Clinical Efficacy Indicators

A total of 8 RCTswere included [8–13, 15, 16], including 393 patients in the treatment group and 396 patients in the control group. After the heterogeneity test (*I*^2^ = 0% < 50%) and *Q* test (*P* = 0.94 > 0.1), indicating that there was no significant heterogeneity among the selected literatures, the fixed effects model was selected for meta-analysis: the clinical efficacy of the observation group was higher than that of the control group (OR = 4.07, 95% CI 2.64-6.27), and the difference was statistically significant (*Z* = 6.38, *P* < 0.00001), as shown in Figure 3.

#### 3.1.2. The Mayo Score

Four literatures [8–10, 13] were included to report the Mayo score, including 385 patients. Meta-analysis was performed to compare the improvement of the Mayo score between the oral vitamin D group and the control group. The MD value was used as the effect scale, and there was no statistical heterogeneity between studies (*I*^2^ = 0%, *P* = 0.82).Our study reveals: (MD: -0.41, CI = [−0.47, −0.34], *Z* = 13.09, *P* < 0.00001). The difference was statistically significant, indicating that oral vitamin D significantly reduced the Mayo score, as shown in Figure 4.

#### 3.1.3. Levels of Inflammatory Factors

A total of 4 literatures [8, 12, 14, 17] measured the improvement of ulcerative colitis by the levels of inflammatory factors (IL-6, TNF-*α*, and CRP). Two literatures [8, 14] included IL-6 and TNF-*α* indicators, and 4 literatures [8, 12, 14, 17] included CRP indicators. Using the MD value as the effect scale, the subgroup analysis showed that the *I*^2^ of the three groups was all less than 50%, showing homogeneity. Using fixed effects model analysis, in the IL-6 group (MD = −4.50, 95% CI (-5.13-3.87), *P* < 0.00001), TNF-*α* group (MD = −7.27, 95% CI (18.96-5.58), *P* < 0.00001), and CRP group (MD = −1.49, 95% CI (-1.76~-1.23), *P* < 0.00001), the differences in the three groups were statistically significant, suggesting that oral vitamin D can effectively reduce the levels of inflammatory factors, as shown in Figure 5.

#### 3.1.4. Intestinal Barrier Function

Four of the included literatures [9, 11, 13, 14] used serum MDA or DAO indicators to describe intestinal barrier function, and MD was used as the effect scale. The results showed that the serum MDA group had homogeneity (*I*^2^ = 0%, *P* = 0.76). The fixed effects model was used for analysis (MD = −0.75, 95% CI (-0.96~-0.53), *P* < 0.00001), and the difference was statistically significant. Heterogeneity was observed in the serum DAO group (*I*^2^ = 81%, *P* = 0.001), and the random effects model was used for analysis (MD = −1.17, 95% CI (-1.39-0.95), *P* < 0.00001). The difference was statistically significant, as shown in Figure 6. Due to the heterogeneity of the 4 studies in the serum DAO group, the remaining 3 studies show homogeneity (*I*^2^ = 26%, *P* = 0.26) after sensitivity analysis and were analyzed using the fixed effects model (MD = −1.00, 95% CI (-1.08~-0.92), *P* < 0.00001), as shown in Figure 7. The difference was statistically significant, suggesting that oral vitamin D improved the repair function of intestinal mucosa in both serum MDA and DAO indexes.

#### 3.1.5. Incidence of Adverse Reactions

A total of 4 studies [8, 11, 12, 16] described the incidence of adverse events, and the heterogeneity test (*I*^2^ = 30% < 50%, *P* = 0.23 > 0.1) suggested that there was no significant heterogeneity among the selected literatures, so the fixed effects model was selected for meta-analysis. There was no statistical significance between the two groups (OR = 0.73, 95% CI (0.34-1.32), *P* = 0.23), as shown in Figure 8. It indicated that there was no significant difference in the incidence of adverse reactions between the oral mesalazine+vitamin D group and the single mesalazine group. However, more literatures may be required to be included in the future to further confirm the reliability of the results due to the small number of literatures included.

### 3.2. Risk Analysis of Bias

The funnel plot was drawn based on the influence of the included literature on the cure rate of UC, and the results showed that the circle was located around both sides of the midline, presenting an incomplete symmetrical distribution, suggesting a large possibility of publication bias in this study, as shown in Figure 9.

## 4. Discussion

### 4.1. Mechanism of Vitamin D Adjuvant Treatment of UC

Vitamin D is a fat-soluble steroid hormone that is mainly present in the human body in two forms: plant-based vitamin D2 and animal-derived vitamin D3, both of which can be ingested through food [20]. Vitamin D is linked to biological processes such as regulating intestinal mucosal immunity and intestinal integrity, in addition to regulating calcium and phosphate metabolism and skeletal homeostasis [21]. Vitamin D insufficiency has thus been linked to immune-mediated illnesses, such as inflammatory bowel disease. Inflammatory response, intestinal microflora disorder, and mucosal barrier damage play an important role in the occurrence and development of ulcerative colitis, and vitamin D can induce and maintain UC remission through reducing inflammatory factors and promoting the repair of intestinal mucosal barrier [22, 23]. In previous systematic reviews, no study evaluated vitamin D as a supplement to adjuvant therapy for UC. In this study, through quantitative synthesis, it was found that compared with the control group, UC patients treated with vitamin D as adjuvant therapy had beneficial effects on the Mayo score, intestinal barrier function, IL-6, TNF-*α*, CRP, and other inflammatory factors. There was no significant difference in safety.

Vitamin D can reduce the levels of inflammatory factors. First, 1,25(OH)2D3 combined with vitamin D receptor (VDR) can induce the expression of anti-inflammatory factors in monocytes to reduce inflammatory factors [24]. Second, vitamin D can act directly on CD4 and T lymphocytes to enhance Th2 cell proliferation and differentiation while inhibiting Th1 cell proliferation in DC cells [25]. Vitamin D can upregulate mitogen-activated protein kinase phosphatase-1 and inhibit the activity of mitogen-activated protein kinase (MAPK) and reduce the production of TNF-*α* while decreasing IL-6 [26]. Multiple studies included in this study showed that vitamin D supplementation effectively reduced the levels of inflammatory factors (IL-6, TNF-*α*, and CRP) in patients with ulcerative colitis. The proposed inflammatory outcome index was consistent with Xue et al. [27]. Xue et al. collected biopsy samples from 103 patients with UC and found that vitamin D/vitamin D receptor (VDR) signaling has a protective effect on the onset or progression of inflammatory bowel disease (IBD) and proved that the activation of hypoxia-inducible factor 1*α* (HIF-1*α*) is closely related to inflammatory factors. HIF-1*α* inhibitors inhibit the expression of TNF-*α*, IL-6, and IL-17, thereby reducing the inflammatory response.

Furthermore, the most prominent pathogenesis of UC is mucosal barrier degradation, which can be separated into mechanical, immunological, chemical, and biological barriers. The four are self-contained and interact with one another, forming a massive defence system against foreign pathogenic pathogens [28]. Vitamin D enhances the connection between intestinal epithelial cells by promoting the expression of transmembrane proteins such as occludin and claudin and mucosal tight junction proteins such as zo-1, zo-2, and zo-3, thus constituting the mechanical barrier of intestinal mucosa [29, 30]. Based on mouse modeling, Wibowo et al. [31] gave different doses of vitamin D on the basis of blank control. By observing the intestinal brush-like margin component protein and the DAO level in peripheral blood under a microscope, it was concluded that vitamin D3 could activate the Wnt protein pathway, thus leading to cell differentiation and proliferation through stem cell signal transduction. Increase the proliferation of colonic mucosa cells to repair the colonic mucosa. Four of the literatures included in this study described intestinal barrier function by serum MDA or DAO indicators. After the mucosal cells of UC patients are damaged, DAO located in the mucous villi falls off and enters the blood and intestinal lumen [32]. When an inflammatory reaction occurs, a significant number of germs and endotoxins enter the bloodstream, and the body goes into survival mode, which inhibits SOD activity, weakens disproportionation reaction, and raises MDA levels as a lipid peroxide metabolic degradation product [33]. Therefore, DAO and MDA levels in peripheral blood are helpful to evaluate the degree of mucosal injury.

Recent studies have found that UC patients may be deficient in trace elements due to intestinal symptoms that lead to reduced nutrient intake and intestinal microbiota disorder, resulting in impaired mucosal barrier [34–36]. Vitamin D deficiency is more common [37]. Horta et al. [38] conducted a prospective study of 44 IBD patients living in Los Angeles (73% of whom had UC) and concluded that 75% of the patients had varying degrees of vitamin D deficiency. Vitamin D can improve intestinal microflora imbalance, regulate immunity, and maintain the integrity of intestinal mucosal barrier, so it is recommended for the treatment or adjuvant treatment of UC. Therefore, this study adopted meta-analysis to analyze the efficacy and safety of vitamin D in the treatment of UC, providing evidence-based medical evidence for the clinical application of vitamin D.

### 4.2. Research Limitations

Studies on vitamin D adjuvant treatment of UC are still in the initial stage. Although meta-analysis showed that vitamin D can improve UC symptoms from repairing the intestinal mucosa and reducing inflammatory factors, there are still many deficiencies. In one thing, the sample size of the literatures included in this study was limited, which was consistent with the small number and low quality of the literatures. This may be because vitamin D has not been unified into the treatment standards in China. I In one thing, In anthor thing, there were some differences in the measurement, usage, and course of vitamin D in the included literatures. In the future, more rigorous and prospective researches will be needed, such as collaboration between multiple centers.

## 5. Conclusion

Meta-analysis results show that, compared with the control group, vitamin D supplement is an effective intervention for UC. Vitamin D supplementation can increase intestinal mucosal repair factors and reduce inflammatory factors and Mayo risk score in UC patients. The results showed that there was no significant difference in the incidence of adverse events between the two methods, and it was a relatively safe adjuvant therapy. Moreover, vitamin D adjuvant therapy has the advantages of simplicity, effectiveness, safety, and low price. However, due to the lack of corresponding multicenter and high-quality RCTs in China and the small number of foreign RCTS, the quality of evidence obtained is not high, and large-sample and high-quality RCTs are still needed to further verify its efficacy. To establish the therapeutic impact and quality of life, more randomised controlled trials with rigorous study design are required, and immune response of vitamin D supplementation in patients with ulcerative colitis and other related chronic complications should be further elucidated.

## Figures and Tables

**Figure 1:** Specific process of literature screening.

**Figure 2:** Risk of bias in the included literature for vitamin D treatment of UC.

**Figure 3:** Forest map of clinical efficacy comparison.

**Figure 4:** Forest map of Mayo score comparison.

**Figure 5:** Forest map comparing inflammatory factors.

**Figure 6:** Forest map of intestinal barrier function comparison.

**Figure 7:** Sensitivity analysis of intestinal barrier function.

**Figure 8:** Forest plot comparing the incidence of adverse reactions.

**Figure 9:** Funnel plot.

**Table 1:** Baseline characterization of included literatures.

Author and year	Case load (T/C)	Gender (male/female)	Age (T/C, year)	Intervening measure	Time (w)	Outcome	Random method
Yu Xia 2020 [9]	60/60	61/59	38.4 ± 3.3 38.2 ± 3.1	C: mesalazine T: mesalazine+VD	8	①②④	—
Senyuan Zheng 2021 [10]	52/51	51/52	39.95 ± 6.5	C: mesalazine T: mesalazine+VD	8	①②	—
Haipeng Dou 2021 [11]	44/44	58/30	46.1 ± 10.7 44.7 ± 8.9	C: sulfasalazine T: sulfasalazine+VD	4	①③④⑧	Random number table
Ningning Yue 2020 [8]	40/40	38/44	41.30 ± 11.16 40.98 ± 10.94	C: mesalazine+placebo T: mesalazine+VD	8	①②⑤ ⑥⑦⑧	Computer stochastic method
Hongliang Gao 2021 [12]	57/59	59/57	40.2 ± 6.30 39.6 ± 6.90	C: mesalazine T: mesalazine+VD	24	①⑥⑨	—
Fenghui Chen 2018 [13]	40/42	44/38	42.30 ± 10.48 43.45 ± 12.5	C: mesalazine T: mesalazine+VD	6	①②③④	Random number table
Rong Yang 2017 [15]	40/40	51/39	41.19 ± 10.23 43.07 ± 11.87	C: mesalazine T: mesalazine+VD	12	①	—
Yang Jing 2019 [14]	99/99	104/94	41.38 ± 5.34 42.35 ± 5.09	C: mesalazine T: mesalazine+VD	4	④⑤⑥⑦	—
Shusheng Zhu 2015 [16]	60/60	60/60	34.6 ± 3.6	C: mesalazine T: mesalazine+VD	4	①⑧	—
Vahedi 2016 [17]	45/45	49/41	37.5 ± 9.0 35.0 ± 9.2	C: mesalazine+NS T: mesalazine+VD	6	⑥	Random number table

T: treatment group; C: control group. Clinical observation indicators: ①—effective rate, ②—Mayo risk score, ③—serum MDA, ④—serum DAO, ⑤—IL-6, ⑥—CRP, ⑦—TNF-*α*, and ⑧—incidence of adverse reactions.

## Data Availability

The datasets used during the current study are available from the corresponding author on reasonable request.
